# A Study Using Power Cycling on the Affective Responses of a Low-Volume High-Intensity Interval Training to Male Subjects with Type 2 Diabetes in Different Physical Activity Status

This article has been retracted.

**DOI:** 10.1155/2021/1255943

**Published:** 2021-11-28

**Authors:** Jun Li, Ruichen Jiang, Wei Cheng, Haifeng Ma

**Affiliations:** ^1^School of Physical Education and Sport Training, Shanghai University of Sport, Shanghai 200438, China; ^2^School of Psychology, Shanghai University of Sport, Shanghai 200438, China; ^3^Department of Endocrinology, Yangpu Hospital, Tongji University, Shanghai 200090, China

## Abstract

High-intensity interval training (HIIT) has been shown in studies to enhance glucose management and cardiovascular well-being in patients with type 2 diabetes. In this study, we used power cycling to assess the physical activity levels of men with type 2 diabetes during a single low-volume HIIT session. First, fifty-six men with type 2 diabetes volunteered to take part in the study, and they were split into two groups based on the International Physical Activity Scale Short Form (IPA). To the first 1–4 labor bouts, both the sufficiently physically active and insufficiently physically active groups exhibited equal positive emotional reactions (*p* > 0.05). However, over time (about 5–10 times), both of them showed reduced emotional reactions, with a significant difference (*p* < 0.01). The insufficiently physically active group had lower mean emotional response, lowest effective response, and maximum effective response values than the sufficiently physically active group (*p* < 0.001), while the difference in RPE between the two groups was not statistically significant (*p* > 0.05). From the standpoint of emotional response, the proposed model shows that HIIT or reduced volume HIIT exercise prescriptions should be utilized with caution in physical activity programs for novices and less active and chronically sick persons. The frequency, intensity, and effects of low-volume HIIT on individuals' emotional reactions and health conditions in the T2DM group are also investigated. Furthermore, this low-volume HIIT program can be successfully applied in the real-world setting of people who are not physically active enough or who are chronically unwell.

## 1. Introduction

Influential activity and arranged exercise therapies can prevent the onset of mental illnesses and have a variety of medical benefits as adjunctive therapy for people with physical and mental illnesses [1–6]. They are also being advocated as an essential component of type 2 diabetic mellitus (T2DM) treatment [7–14]. Several recent studies have looked at the influence of real idleness on the progression of T2DM, which is considered a risk factor for the progression of T2DM [15–20]. Furthermore, higher levels of actual employment and exercise may reduce the risk of T2DM and certain comorbidities, as well as improve patient's side effects and quality of life (QoL) [21]. However, suggestions for focused energy practice treatment in individuals with T2DM are hampered by the fact that it is considered excessively extreme and aversive for individuals who are inactive and additionally at risk of ongoing infections, and thus less likely to cling to it [22, 23]. In the T2DM population, high-intensity interval training (HIIT) is characterized by brief. Intermittent vigorous activity interspersed with rest or low-intensity exercise, as opposed to high-intensity continuous exercise with regular rest periods, and it is a more viable alternative to high-intensity continuous exercise and moderate-intensity continuous training. For individuals with T2DM, this is a more feasible option to high-intensity continuous exercise and moderate-intensity continuous training, producing equal or even greater benefits on physiological changes and health-related markers [24–26]. However, most “all out” HIIT or sprint interval training (SIT) needs specialized equipment [27] and high levels of desire that may not be safe or feasible for the physically inactive T2DM population [28–30], implying that these training modalities will have a significant detrimental impact and are likely to have severe negative effects and cause avoidance reactions during exercise treatments.

On the other hand, as previously reported in observational studies [17, 31], feelings of pleasure during exercise are determinants of participation and persistence. Therefore, exercise prescriptions that enhance the acquisition of pleasurable sensations can contribute to positive benefits for subjects in terms of maintenance of exercise and health. Considering that the characteristics of HIIT are based on the individual cardiorespiratory fitness of the subject, that intensity is not standardized, and that the majority of the T2DM population is overweight (obese), physically inactive, and lacking in time, it means that HIIT training programs can be individualized and do not have to involve “all out” HIIT or SIT [32]. Low-volume HIIT, which involves a fairly low total exercise volume and time, has similar effects on glycaemic control to those observed with high-volume exercise [13] and can cause rapid improvements in cardiovascular and metabolic health. Considering that lack of time and rejection of longer, high-intensity training are barriers to regular exercise participation [33, 34], there is a need to develop effective and health-promoting low-volume HIIT exercise prescriptions in the T2DM population [29, 35–37]. It has been shown that active subjects report more positive affective responses (pleasure) than sedentary subjects during moderate-to-high-intensity exercise [38–42]. However, these studies have compared the affective responses of subjects during a continuous exercise regimen and have not compared affective responses during a single session of low-volume HIIT in T2DM subjects with different physical activity states [43].

In this paper, we aimed to apply power cycling to affective responses before-mentioned those pleasurable and unpleasant feelings. HIIT protocol was provided to male subjects with T2DM of modifying physical activity status to a single session of a low volume. The proposed model that was sufficiently physically active would have a more pleasant emotional response to a single low-volume HIIT exercise than people who were not enough physically active. The low-volume HIIT protocol, which used power cycling as the apparatus, consisted of 10∗60 seconds of exercise at 90–95 percent of maximum heart rate, followed by 60 seconds of active recovery at 25–30 percent of maximum heart rate, with affective responses (sensory scale, −5/+5) and Borg's RPE 6–20 scale (Borg's Rating of Perceived Exertion) recorded in the final 10 seconds of each high-intensity session. Independent samples *t*-tests, two-factor repeated-measures ANOVA, and chi-square tests were used to evaluate the data. In addition, measuring both perceived intensity and affective variables during a single bout of vigorous exercise can determine the physiological and psychological benefits of exercise prescriptions.

The rest of the paper is organized as follows. In Section 2, materials and methods of the proposed model are described. The performance measures are further summarized in Section 3. Statistical analysis is discussed in Section 4.  Section 5 discusses experimental results and performance evaluation.  Section 6 gives a detailed discussion on results. Finally, Section 7 concludes the paper with a summary and future research directions.

## 2. Materials and Methods

### 2.1. Benchmark Dataset

The study protocols and possible risks were thoroughly discussed to the individuals before the study, and signed informed consent was acquired from all subjects. The study protocol was approved by the local hospital's ethics committee (ethics committee protocol number) (LL-KY-009). Before the study, all participants filled out a medical history questionnaire, the PAR-Q, and the International Physical Activity Abbreviated Questionnaire (IPAQ-SF) at a hospital in Shanghai's Yangpu District as shown in Table 1. The inclusion criteria given below were used to select 56 participants.

#### 2.1.1. Physical Examination

Physical examination included diagnosis of T2DM for at least one year, meeting WHO diagnostic criteria for diabetes [44], no major macroscopic or microscopic vascular complications of diabetes; age 25 to 60 years; body mass index (BMI) <35 kg/m^2^, body mass index calculated as weight divided by height squared. There are no physical limitations to the exercise intervention to be performed and no major health problems.

#### 2.1.2. Behavioral Habits

Behavioral habits included no smoking in the past 6 months, no participation in a supervised exercise program, and maintenance of a diet for at least 6 months.

#### 2.1.3. Exercise Testing

Prior to participation in the trial, all participants underwent a detailed medical evaluation to screen for relative or absolute contraindications to high-intensity exercise, including using the Bruce protocol for exercise panel testing to confirm the absence of potential cardiac contraindications.

#### 2.1.4. Exclusion Criteria

Exclusion criteria included medical conditions that precluded exercise; participants receiving exogenous insulin therapy; smokers; unstable weight with evidence of acute disease, renal, hepatic, or cardiovascular disease; changes in dietary patterns; nonperformance of all experimental requirements; and participation in other supervised exercises.

### 2.2. Methodology

The participants were divided into two groups based on their level of physical exercise: those who were physically active enough (*n* = 28) and those who were not active enough (*n* = 28), with each participant going through the following procedures. Both groups received instruction from a fitness instructor. First and foremost, a physical examination and screening are required. Then, there is exercise testing, followed by a single low-volume HIIT workout. One supervised low-volume HIIT session on a Swedish Monark power bicycle, using an effective response and Borg's RPE scale in front of the power bicycle and monitored with a heart rate band (polar). This was a single trial with repeated measurements in two subject groups designed to compare the affective responses of T2DM subjects with different physical activity states during a single session of low-volume HIIT.

One week prior to the start of the study, subjects were given a tour of the laboratory and power bicycle and a detailed explanation of the procedure, an introduction to the specified low-volume HIIT, a request for a maximal exercise test, and a low-volume HIIT adaptation, starting at a lower speed and load and progressing to the experimental intensity as the patient was able to tolerate. Subjects in both groups received three 15-minute behavioral counseling sessions (45 minutes total) in the week prior to the trial, with the goal of gradually increasing the load via power bicycle to achieve the intensity tested in the study, one-on-one counseling to prepare subjects for transition to an exercise prescription, and standard counseling on topics such as nutrition or exercise, including overcoming barriers to exercise, enhancing self-regulation, self-efficacy, and increasing awareness of the physical and mental benefits of exercise to improve trial compliance. During the study period, participants also received information on maintaining activities of daily living (daily diet, habitual physical activity, and medication), considering that fluctuating blood glucose levels may be more harmful than high and stable levels, and all subjects were monitored on a 14-day real-time blood glucose monitor for the first two weeks to avoid excessive fluctuations in blood glucose. Before the exercise experiment, patients were given a detailed explanation of the Feeling Scale of Affective Responses (FS), the RPE scale, and their meaning, and they were given a preexperimental adaptation process to familiarize themselves with the forms and the experimental procedure.

## 3. Performance Measures

### 3.1. Assessment of Physical Activity Level

The order of actual work status depended on the ACSM rules [30], utilizing an abbreviated form of the International Physical Activity Questionnaire (IPAQ) [45–47]. In the first place, subjects were gotten some information about their actual work seven days sooner yet additionally about their actual work design during the past 90 days, that is, their actual work status during ordinary life. The inadequately genuinely dynamic gathering included <150 minutes of actual work each week and <75 minutes of moderate-power and did not take part in any ordinary actual work, while the adequately truly dynamic gathering met no less than either of these rules, routinely performed non-serious exercise, obstruction preparing, and vigorous exercise, and knew about span preparing; yet none of the subjects in either bunch had related knowledge to the HIIT convention utilized in this investigation of the program.

### 3.2. Exercise Test

All subjects had previous experience with outdoor bicycle, but pretraining was required for power bicycle balance and leg exertion. Heart rate (beats/minute) was recorded continuously throughout the test wearing a Polar heart rate monitor. Heart rate should reach 90–95% × (220- age) of the predicted maximum HR during high-intensity training, and Borg's RPE scale [48] was used to assess whole-body subjective exertional sensations during each round of the low-volume HIIT protocol of the maximal exercise test, with all participants receiving Borg's RPE scale standardized for use prior to testing [49].

### 3.3. Borg's RPE Scale

Borg's RPE scale was used to assess HIIT in the return of whole-body motor perception. Prior to the exercise test, the meaning of self-perceived movement was explained to the subject. The minimum exercise intensity on Borg's RPE scale was 6 (rest), and the maximum exercise intensity was 20 (exhaustion). The RPE value is recorded at the last 10 seconds of each minute of the HIIT high-intensity sprint.

### 3.4. The Feeling Scale for Affective Responses (FS)

FS is an 11-point biphasic scale ranging from −5 to +5 and is commonly used to measure affective responses (happy/unhappy) during exercise [50–52]. This scale presents the following linguistic orientations: −5 = very bad; −3 = bad; −1 = bad; 0 = neutral; +1 = OK; +3 = good; +5 = very good, and previous studies have suggested the use of this scale to measure affective responses during exercise [30, 39, 41, 43, 51]. A copy of the FS was applied. and FS values were recorded during the last 10 seconds of each high-intensity sprint during the low-volume HIIT implementation.

### 3.5. Low-Volume HIIT Exercise Program

Heart rate was continuously monitored throughout the supervised exercise intervention to provide a basis for the number of repetitions and duration of each repetition to ensure that the subject was training at the desired intensity training. During exercise, when the heart rate rose too rapidly, the researcher made inquiries and stopped the experiment immediately if there was discomfort. If chest tightness, heart pain, or headache was observed, the experiment was stopped immediately, and participants were allowed only simple household chores, walking, and other daily physical activities before the exercise intervention, except for adaptation to the low-volume HIIT exercise protocol.

Prior to the implementation of HIIT, subjects progressively performed a 5-minute warm-up at less than 50% intensity. HIIT consisted of 10 sets of 60 seconds of work at 90–95% of intensity and 60 seconds of active recovery at 25–30% of intensity. This low-volume HIIT model, adapted from Gibala et al. [8], is suggested as a feasible and tolerable exercise prescription for both healthy and clinical populations. The HIIT protocol, including warm-up and cool-down, was completed in 30 minutes, with the last 10 seconds of each high-intensity sprint, as reported by the subjects (Borg's RPE scale, 6–20) and affective response (FS, −5/+5), and the order of presentation of Borg's RPE scale and FS was randomized. The duration of each exercise session (minutes) was allocated as follows: 5 minutes of warm-up (first 3 minutes off-bicycle, second 2 minutes on-bicycle, heart rate in the 90–95% range) and 20 minutes of HIIT per session: 10 minutes at 90–95% intensity, 9 minutes of interval active recovery at approximately 25–30% intensity, and 5 minutes of relaxation and finishing (see Figure 1).

## 4. Statistical Analysis

The information was communicated as mean and standard deviation (SD), and the Shapiro-Wilk strategy was utilized to test for ordinariness, and free examples *t*-tests were utilized to analyze the qualities of subjects between gatherings, just as the mean, greatest, and least emotional reactions during the HIIT test, and the full of feeling reactions at the most extreme RPE. Cohen's *d* was utilized to compute impact sizes for these examinations. A two-factor bunch blended model rehashed measures ANOVA investigation was utilized to think about full of feeling reactions and RPE between the two gatherings of subjects in the low-volume HIIT. At the point when the sphericity supposition was abused, the Greenhouse-Geisser épsilon revision is prescribed to decide the impact sizes for these examinations utilizing the one-sided estimated time of arrival square (*η*^2^*p*), and LSD post hoc test is utilized to figure out where critical contrasts happen. A chi-square test was utilized to analyze the frequencies of positive and negative full of feeling reactions toward the start (work adjusts 1–3), center (work adjusts 4–7), and end (work adjusts 8–10) of the two HIIE adjusts and to confirm potential contrasts in the dissemination of subjects with good or negative mean FS scores in each gathering, who were ordered as disagreeable HIIT and lovely HIIT. Pearson connection coefficients were utilized to test for potential connections between emotional reactions and RPE reactions in the two gatherings. For the investigation, the importance level was set at 5% (*p* < 0.05) and all information was broken down utilizing SPSS 25.0.

## 5. Experimental Results

As illustrated in Figure 2, subjects underwent a low-volume HIIT program, which elicited an emotional response. The subject count effect yielded *F* = 151.238, *p* 0.001, 2*p* = 0.967, while the group interaction for time yielded *F* = 17.032, *p* 0.001, 2*p* = 0.769. Post hoc analysis using LSD revealed that the insufficiently active group had lower emotional reactions on work rounds 5–10 than the adequately active group (*p* 0.001), as revealed by the group interaction (*F* = 40.418, *p* 0.001, 2*p* = 0.428). Only on the ninth time did the adequately engaged group show reduced emotional reactions.

Inactive and inadequately active men's emotional responses following a single session of high-intensity interval exercise are shown in Table 2, with the mean (*p* < 0.001), lowest (*p* < 0.001), and greatest (*p* < 0.001) emotional reaction values. In the insufficiently active group, the maximum RPE emotional responses were lower than in the properly active group. Furthermore, the group that was not adequately active had a greater proportion of participants categorized as uncomfortable HIIT subjects.  Table 3 shows a higher frequency of negative emotional reactions in the middle of the low-volume HIIT regimen.

For positive/neutral affect, Feeling Scale values ≥ 0; for negative affect, Feeling Scale values = 0. Within-subjects count effect findings for degree of subjective exertion in the HIIT protocol indicate *F* = 992.403, *p* 0.001, 2*p* = 0.995, where the group interaction for count shows *F* = 4421.959, *p* 0.001, 2*p* = 0.988. Similarly, the between-group interaction (*F* = 505.421, *p* 0.001, 2*p* = 0.990, post hoc analysis using LSD showing no statistical difference in the degree of subjective exertion relative to the active group) as shown in Figure 3 revealed no statistical difference in the degree of subjective exertion relative to the active group. Insufficiently active males with T2DM exhibited poorer effective responses, but similar to the adequately active group RPE, the same results were obtained in the previous continuous exercise program, with a strong negative connection between the two, regardless of physical activity status (Figure 4).

## 6. Discussion

In this research, a low-volume HIIT program was coordinated on male subjects with type 2 diabetes using a power bicycle, a common contraption in genuine wellbeing, and recuperation settings, considering Gibala et al. [8, 53, 54]. Gibala et al. proposed a low-volume HIIT program for the T2DM people. It has been suggested that it very well may be an incredible framework to redesign physiological limits and hinder cardiometabolic infection in T2DM people. Similarly, the loaded feeling responses to the execution of this action program in the T2DM people have been less generally thought of. Enough powerful assembling had an all the more sure loaded with feeling response to low proportions of HIIT than the inadequately unique social event [55]. The key finding was that the two social occasions reflected correspondingly at the completion of the underlying four low-volume HIIT gatherings. Additionally, the inadequately unique social affair showed a negative enthusiastic response after some time during the low-volume HIIT show. Brimming with feeling response lessened with growing activity length and repeat in the two social events (e.g., Figure 2 and Table 2). It has been shown that there is a negative connection between movement power and joy, with training power over the ventilatory edge (close to the respiratory compensation point) making homogeneous horrendousness [22, 56]. The inadequately powerful assembling point by point enterprising palatability in the second half of the HIIT is unmistakable. The fifth rep on the power bicycle, however, in the sufficiently unique social event showed a similar response exclusively after the eighth [57, 58].

Moreover, it was seen in the review that there were still a few subjects from the adequately dynamic gathering who saw the low measure of HIIT as lovely stages 1–3 (85.7%), 4–7 (32.1%), and 8–10 (2.4%), though a few people from the dynamic gathering saw the low measure of HIIT as disagreeable stages 1–3 (3.6%), 4–7 phases (35.7%), and even as high as (81%) for stages 8–10 (Table 3). Hence, subjects' activity inclinations or character variables might be very heterogeneous concerning passionate reactions in HIIT, for example, earlier exercise insight and knowledge of activity designs, which can to a great extent impact the intellectual cycles engaged with creating enthusiastic reactions to practice [41, 59], and absence of HIIT experience can bring about people encountering more negative passionate reactions. The adequately dynamic gathering in the current review, albeit not presented to formal HIIT, may likewise have had earlier exercise insight and knowledge of activity designs and additionally practice regimens that fundamentally impacted full of feeling reactions to HIIT. Notwithstanding, further exploration proof is as yet deficient. In this sense, examine which mental variables might be identified with the full of feeling reaction to HIIT. Further examination of information on practice inclination, inspiration, and character would be useful, particularly in the T2DM populace, where the inspiration to practice is especially significant. It is likewise conceivable that over the long run, the inconvenience felt by the inadequately dynamic gathering is related to exceptionally engrossed considerations and less fortunate self-adequacy.

Thus, during continuous HIIT, less active subjects had reduced emotional responses over time [60–62] and may have approached heavy workloads more negatively. For overweight/obese underactive subjects, HIIT protocols longer than 120 seconds are perceived as unpleasant [63–65], and similar results were found for low-volume HIIT and affective responses decreased over time. Lunt et al. [66] demonstrated that, compared to moderate-intensity continuous exercise, subjects trained in real-world HIIT-trained subjects showed modest improvements in cardiorespiratory fitness. The main reason for this finding is related to reducing adherence to the HIIT program.

Few studies have studied the emotive reaction to each stroke of HIIT too far, and the results have been inconsistent [57, 65, 67, 68], particularly in the T2DM group, where there is less specific testing of the affective response to low-volume HIIT. Given that the majority of T2DM patients are sedentary or inactive, these findings may be useful in terms of public health. (1) The participants' physical activity status was not directly measured; instead, we used a questionnaire, which may underestimate or overestimate the subjects' current level of physical activity; (2) it should be noted that the T2DM population differs from the general population in that cardiorespiratory fitness and physical activity are generally low, but (3) there is insufficient evaluation of individuals' mental condition, and further study is needed on affective reactions during low-volume HIIT.

## 7. Conclusions

Exercise is an important component to complement daily physical inactivity and to combat T2DM. It is considered an important tool in the prevention and management of T2DM and its complications, including glycaemic control, cardiometabolic risk, and mental health. The overall performance of the proposed model shows that the insufficiently active group reported pleasurable feelings during sessions 1–4 and the sufficiently active group reported pleasurable feelings during sessions 1–8, but both affective responses became more unpleasant with time and the number of high-intensity interval sprints. Moreover, it is recommended that HIIT or lower volume HIIT exercise prescriptions should be used with caution in physical activity programs for beginners and less active and chronically ill individuals from affective response perspective.

In the future, a new maturity level will be introduced, as well as individuals who are less active and inexperienced with suprathreshold exercise intensities are required to investigate HIIT. It is crucial to note that HIIT's acceptance and practicality are still in their early stages, requiring more research.

## Figures and Tables

**Figure 1:** Low-volume HIIT.

**Figure 2:** Affective responses during a single bout of high-intensity interval training in active and insufficiently active group. ^∗^Different from the insufficiently active group (*p* < 0.05).

**Figure 3:** Rating of perceived exertion during a single bout of high-intensity interval exercise in active and insufficiently active men.

**Figure 4:** Correlation analysis between affective response and rating of perceived exertion during a single bout of high intensity.

**Table 1:** Basic characteristics and data of subjects (IPAQ: International Physical Activity Questionnaire).

Characteristics	Active (*n* = 29)	Insufficiently active (*n* = 29)
Age (years)	39.2 ± 4.3	40.5 ± 5.1
Height (cm)	173.7 ± 6.6	172.9 ± 6.2
Weight (kg)	74.76 ± 8.96	75.81 ± 9.06
Body mass index (kg/m^2^)	25.98 ± 5.02	26.75 ± 4.22
Maximal heart rate (bpm)	179 ± 8	177 ± 7
Diagnostic time (years)	1.84 ± 0.49	1.95 ± 0.55

*IPAQ score (MET.min.wk* ^*−1*^)		
Walking	228 ± 202^*∗*^	131 ± 80
Moderate physical activity	1102 ± 436^*∗*^	252 ± 121
Vigorous physical activity	896 ± 728^*∗*^	128 ± 115
Total physical activity	2226 ± 798^*∗*^	511 ± 72

^*∗*^Statistically significant compared with the insufficiently active group **(***p* < 0.05**)**.

**Table 2:** Mean affective response, lowest affective response, highest affective response, and affective response in the highest rating of perceived exertion during a single bout of high-intensity interval exercise in active and insufficiently active men.

Variables	Active (*n* = 29)	Insufficiently active (*n* = 29)	ES
Mean affective response	1.43 ± 2.10^*∗*^	−1.15 ± 1.39	1.45
Lowest affective response	−0.64 ± 1.63	−2.34 ± 2.32	0.85
Highest affective response	2.07 ± 1.80^*∗*^	1.19 ± 1.81	0.49
Affective response at the highest RPE	−0.4 ± 1.53	−1.36 ± 2.20	0.51

^*∗*^Different from the insufficiently active group (*p* < 0.01); ES = effect size.

**Table 3:** Frequency of the positive/neutral and negative affective responses in the beginning, in the middle, and in the end of the high-intensity interval exercise in insufficiently active and active men.

Work bouts	Positive/neutral affect		Negative affect	
	Active	Insufficiently active	Active	Insufficiently active
1–3	81 (96.4%)	72 (85.7%)	3 (3.6%)	12 (14.3%)
4–7	72 (64.3%)	36 (32.1%)^*∗*^	40 (35.7%)	76 (67.9%)^*∗*^
8–10	16 (19%)	2 (2.4%)	68 (81%)	82 (97.6%)

^*∗*^Different from the insufficiently active group (*p* < 0.001).

## Data Availability

All the data used in this study are available from the corresponding author upon a reasonable request.
